# Ethnobotanical Study of Traditional Medicinal Plants Used to Treat Human and Animal Diseases in Sedie Muja District, South Gondar, Ethiopia

**DOI:** 10.1155/2022/7328613

**Published:** 2022-09-19

**Authors:** Amare Bitew Mekonnen, Ali Seid Mohammed, Abeba Kassa Tefera

**Affiliations:** Bahir Dar University, Department of Biology, P.O.Box 76, Bahir Dar, Ethiopia

## Abstract

A variety of traditional medicinal plants has been widely used by different indigenous people in Ethiopia for many human and livestock ailments. This study was conducted to investigate and document the use of medicinal plants in the Sedie Muja district. Sixteen key informants were selected purposively and 72 informants were selected randomly from 5 wards. Data were collected using semi-structured questionnaires, group discussions, and field observation. Besides descriptive statistics, the data were analyzed using some ethnobotanical analysis tools like preference ranking, paired comparison, direct matrix ranking, informant consensus factor, and fidelity level index. A total of 89 species of medicinal plants were identified and collected with 82 genera and 44 families. Out of these, 60 species (67.42%) were used against human ailments, 10 species (11.24%) were used against livestock ailments, and 19 species (21.34%) were used to treat both human and livestock ailments. Herbs constituted the largest growth habit (40 species) followed by shrubs (33 species). The most frequently used plant part was leaves (39.9%), followed by roots (23.83%), and the condition of preparation was fresh plant materials (70.98%). The most widely used method of preparation was crushing (22.8%) followed by crushing-squeezing (11.39%). The most common route of administration was oral (49.74%) followed by dermal (30.05%). *Ruta chalepensis* was the predominant medicinal plant cited by most of the informants 62 (70%) followed by *Ocimum lamiifolium* 59 (67%). The disease category with the highest ICF value (0.90) was the evil eye. There was a high preference for *Euphorbia abyssinica* to treat stomachache. *Ocimum lamiifolium* was the most preferred species for the treatment of febrile illness. Anthropogenic factors are the major threats to medicinal plants. In general, the study area is rich in medicinal plants that have a significant role in the management of various human and livestock diseases.

## 1. Introduction

Ethnobotany is the study of interrelations between humans and plants, including plants used as food, medicines, and for other economic applications [1]. One of the aims of ethnobotanists is to explore the importance of plants that are used as food, clothing, shelter, fodder, fuel, furniture, and medicinal use [1]. Therefore, ethnobotanical studies are useful in identifying, disseminating, and documenting indigenous knowledge and the application of plant diversity for human and livestock ailments [2]. Traditional medicine has been defined as health practices, approaches, knowledge and beliefs in plant, animal, and mineral-based medicines, spiritual therapies, manual techniques and exercises to treat, diagnose and prevent illness or maintain wellbeing [3]. Traditional medicine is the main source to treat both human and livestock diseases which still play a vital role to cover the basic health needs in developing countries [4]. This is because the use of medicinal plants has much lower cost than modern public health services and it is a culturally linked tradition [5].

Trends in the use of traditional and complementary medicine are increasing in many developed and developing countries. According to [6], traditional remedies are the most important and sometimes the only source of therapeutics for nearly 80% of the worldwide population. For instance, about 85% of world population uses herbal medicines for prevention and treatment of diseases and the demand is increasing in developed and developing countries [7, 8]. About 500 million people in south Asian countries alone are reported to seek health security from plants [9]. In Africa, more than 80% of the population uses traditional medicine for their health care practices [3].

Traditional medicine remains the main source for a large majority of people in Ethiopia, about 80% of the human population and 90% of livestock depend on traditional medicines treating health problems [10, 11]. Ethiopia is a home of diversity, having diverse flora as well as ethnic groups, each having different ways of utilization and manipulation of medicinal plants. In addition, the people of Ethiopia have many languages, cultures, and beliefs, which have in turn contributed to the high diversity of traditional knowledge and practices of plant resource uses, management, and conservation [7, 8]. The Ethiopian people use traditional medicine over the past period and categorize plant species indigenously [12]. However, the indigenous knowledge about traditional medicinal plants is transferred secretly from generation to generation orally in developing countries like Ethiopia. Therefore, there were many misconceptions on the efficacy of medicinal plants because of lack of interest of modern society and way of knowledge transfer by elders [13].

The traditional medicine in Ethiopia is facing a problem of sustainability due to loss of taxa, loss of habitat, and loss of indigenous knowledge. The plant species reduced extremely because of environmental degradation, agricultural expansion, loss of forests and woodlands, over-harvesting, fire, overgrazing, firewood collection, and urbanization appear to be the major threats to the medicinal plants of Ethiopia [14]. These factors require urgent attention, to conserve and optimize the use of medicinal plants in primary health care systems of humans and livestock. Moreover, The indigenous knowledge of medicinal plants is getting lost due to migration from rural to urban areas, industrialization, rapid loss of natural habitats, and changes in life style [15]. As a result, the documentation of traditional use of medicinal plants is important to preserve the indigenous knowledge. Therefore, the main objective of this study was to identify the major types of medicinal plants used to treat both human and livestock disease, to document indigenous knowledge, and to identify major threats and conservation methods to keep the balance between availability and utilization of traditional medicinal plants by the community in the Sedie Muja district.

## 2. Materials and Methods

### 2.1. Description of the Study Area

The study was conducted in the Amhara Region, South Gondar zone in Sedie Muja district. The district has 21 kebeles of which 19 rural and 2 urban. Robit is the capital city of the district which is 774 km far from Addis Ababa and 207 km from Bahir Dar. Geographically the district is situated between 11°30′ 0″ North Latitude and 38°30′ 0″ East Longitude (Figure 1). The altitude of the district ranges from 1500 to 2900 meters above sea level (masl). The district has three climatic zones; these are 11% highland, 41% midland, and 48% low land. The primary wet season extends from April to October; among these, July and August are the wettest months. The mean annual rainfall is 1000–1500 mm and the mean annual temperature is 16°C–24°C [16].

The total population of the district is 116,525, of which 55,605 are males and 60,920 are females [16]. According to [16], the number of livestock found in the study area was cattle 68,008, sheep 39,193, goats 55,130, donkeys 12,316 and others. The major common human diseases found in the district include malaria, acute respiratory disease, diarrhea, skin disease, eye disease, tonsillitis, wound, and other infectious and parasitic diseases. These diseases mostly affect people living in the rural areas where the health services are in shortage, they are unable to afford the high cost of modern drugs and are far from the health center [16]. Animals have also suffered from the most common diseases in the Sedie Muja district which include black leg, anthrax, pasturalisis, and salmonellosis, rabies, lumpy skin disease, sheep and goat pox, Newcastle, dermatophytosis, trypanosomiasis, and other parasitic diseases [16].

### 2.2. Selection of Study Sites and Informants

Five kebeles were selected purposely for ethnobotanical data collection based on vegetation distribution, altitudinal range, availability of traditional healers and recommendation from, local authorities, and developmental agents. The 5 selected kebeles such as Ziwa, Gedam Mikael, Anfargie, Keta, and Tara Arbatu (Figure 1) cover the three agro-climatic zones.

A total of 88 informants (33 females and 55 males) between the age of 22 and 85 were selected randomly by lottery method from the local people following [2]. From these informants, 16 key informants were purposely selected based on recommendation from local administrators, health extension workers, and around 3–4 key informants were selected per each 5 kebeles. The equation: *N* = *Z*2 *P* (1−*P*)/C2 is used to determine the number of informants, where “N” is the sample size; “Z” is the standard normal value at 95% of confidence level (i.e., *Z* = 1.96); “*P*” is the proportion of households practicing traditional medicine; and “C” is the marginal error. Therefore (*P*=0.5) at 5% marginal error (*C* = 0.05) and 95% confidence interval.

### 2.3. Data Collection Methods

Ethnobotanical data were collected from March to August 2020. These data were collected using semi-structured questionnaires, field observation, and group discussion. Data of indigenous knowledge on the uses and application of traditional medicine and the threats and conservation status of medicinal plants were collected. According to [2] and [17], ethnobotanical information like the use of these plants to treat common human and animal diseases, methods of preparation, condition of preparation, ways of application, dosage, routes of administration, conservation, and threats of medicinal plants were collected.

Field observations were also conducted in areas where most of the medicinal plants are grown or cultivated. This method was used to obtain actual information from the informants about identification (species local names, habit, and habitat), distribution, conservation status, and threats of medicinal plants.

According to [2], group discussions were briefly conducted at each kebele with 5–7 informants and residents in seeking the traditional medicinal system of the people and its management and to know how knowledge is maintained and transferred from one generation to other generations. Discussions took place based on the checklist of questions such as use, major threats, status of availability, strategies they use for the conservation of medicinal plants, and uses of the plants other than medicine and related data were recorded.

### 2.4. Medicinal Plant Specimen Collection and Identification

Medicinal plant species which were not identified in the field were pressed and dried for voucher specimen to be identified in Ethiopian national Herbarium in Addis Ababa University or by comparing published volumes of flora of Ethiopia and Eritrea edited by [18, 19], and [20]. Some of these medicinal plants' images were collected for further identification (Figure 2).

### 2.5. Data Analysis

The data were analyzed and summarized by descriptive statistical analysis by using Microsoft Excel spreadsheet software. The data were also analyzed by some ethnobotanical analysis tools including informant consensus factor (ICF), preference ranking, paired comparisons, direct matrix ranking, and fidelity level index (FL) techniques.

#### 2.5.1. Informant Consensus Factor (ICF)

According to [2], informant consensus factor was used for categories of diseases to identify the agreement of informants on the reported cures for the group of diseases.

The ICF was calculated as follows: ICF = Nur–Ns/(Nur – 1) Where Nur is the number of use reports from informants for a particular plant-usage category and Ns are the number of species that were used for the plant-usage category. The factor provides a range of 0 to 1, where a high value acts as a good indicator for a high rate of informant consensus.

#### 2.5.2. Preference Ranking

A preference ranking was conducted following [2] to determine the most preferred medicinal plant by key informants report. Accordingly, eight key informants were purposively selected for ranking seven most important traditional medicinal plants that can treat stomachache. Informants identify the best-preferred medicinal plant species for treatment of stomachache. Each informant was expected to assign the highest value (seven) for plant species most preferred, against this illness and the lowest value (one) for the least preferred plant and in accordance of their order for the remaining ones. Then values were summed up and ranks were given to each plant species.

#### 2.5.3. Paired Comparisons

Paired comparisons to indicate the efficacy and popularity of five medicinal plant species used to treat febrile illness were employed as described by [2]. A list of the pairs of selected items with all possible combinations was presented to the selected informant and their responses were recorded and total value was summarized. The number of pairs are calculated by the formula, *n* (*n*−1)/2, where *n* is the number of items. An item with highest frequency of choices has the highest score.

#### 2.5.4. Direct Matrix Ranking

Direct matrix ranking method was used for commonly reported multipurpose medicinal plants to assess their relative importance to the local people and the extent of the existing threats related to their use values following the method of [2]. Six most widely utilized multipurpose plant species and eight use values of these plants were selected and identified. Five selected key informants were allowed to give status of use (5 = best, 4 = very good, 3 = good, 2 = less used, 1 = least used, and 0 = not used). Then use values of each species were taken and the values of each species were summed up and ranked.

#### 2.5.5. Fidelity Level Index

Fidelity level (FL) was calculated for each medicinal plant reported to be used against human and livestock diseases to estimate its relative healing potential using the formula below. FL (%) = (Np/N) *x* 100. Where Np is the number of informants that claim the use of a plant species to treat a particular disease and N is the number of informants that use the plants as a medicine to treat any disease as stated by [2].

## 3. Results and Discussion

### 3.1. Distribution and Diversity of Medicinal Plants of the Study Area

A total of 89 medicinal plant species belonging to 82 genera and 44 families were identified and documented from the study area. Among these, the family Asteraceae constituted the highest number of medicinal plant species 8 (8.9%) followed by Solanaceae and Fabaceae 7 (7.9%) species each. Family Aloaceae contributed the least that constituted only 1 species (Table 1). The families had shown the presence of high utilization of various medicinal plants for health care system in the study area. This result agrees with the finding of [21–23], and [24] in which Asteraceae is the dominant family and the study area is relatively richer in medicinal plant species.

#### 3.1.1. Habitat of Medicinal Plants in the Study Area

Residents of the Sedie Muja district collect and prepare medicinal plants from different habitats. Most of the medicinal plants in the district 53 (59.55%) inhabited in the wild and 29 (32.58%) in home garden and 7 (7.87%) were found both in the wild and home garden. This evidence indicates that the residents mostly depend on medicinal plants inhabited in the wild to prepare remedies in the study area. Moreover, the local people's potential and ability to cultivate around their home garden is mostly very low. According to [12, 15, 25, 26] and [8] explanation, it can be confirmed that the majority of the medicinal plants are found in their wild habitat.

#### 3.1.2. Habit of Medicinal Plants in the Study Area

Medicinal plants that were collected in the district have different habit or growth forms. From the recorded plant species, herbs 40 (44.94%) were the leading growth habit in the study area followed by shrub 33 (37.08%) and tree 8 (8.99%). Very few numbers of medicinal plants have growth form of climbing 8 (8.99%) (Figure 3). This result showed that the most widely used medicinal plants habit in the study area were herbs followed by shrubs. This is because the local communities simply get the herb species plant and the plant species were found high in number in the study area. A similar result was found and the above idea was supported by the findings of [23, 24, 27, 28], and [8]. On the contrary, other researchers such as [29] showed that shrubs were the abundant growth form.

### 3.2. Plant Parts Used

The society uses different parts of the plant for medicinal purposes. The local communities mostly used leaves which 77 (39.9%) followed by roots 46 (23.83%), seed 26 (13.47%), latex 12 (6.22%), stem 9 (4.66%) and others (Table 1). This result showed that leaf is the most commonly used plant part in preparation of remedies. The reason is, it is easy for preparation and collection. However, harvesting the root causes loss of the whole plant since physiological activities are stopped. This finding agrees with the results of other ethnomedicinal studies by [10, 22, 24, 30], and [31] who reported that leaves were the most cited plant part used in remedy preparations. On the other hand, the work of [28, 32], and [33] showed that the root was a widely used plant part.

### 3.3. Methods of Preparation

Regarding to the preparation of traditional medicine, the local people apply various methods of preparations of traditional medicines for different types of ailments. The preparations vary based on the type of disease treated and the actual site of the ailment. The result of this study revealed that the highest proportion of preparations of ethnomedicinal plants employed is by crushing 44 (22.8%), crushing and squeezing 22 (11.39%), pounding and powdering and unprocessing 18 (9.33), powdering 15 (7.78%), concoction 14 (7.25%), squeezing 12 (6.23%), and others. To give immediate response for the diseases and recover from illness, the society mostly applies the method of crushing to extract the bioactive elements of the plant part. Majority of the remedies were prepared using a single plant part of the same plant and few remedies are prepared mixtures of different organs of the same plant or mixture of organs from different plants in the study area. This result is agreed with the findings of [22, 27, 34], and [26] who reported that crushing was the most dominant method of remedy preparations.

### 3.4. Solvents and Additives

The local people use some other products as additives in their preparations. These are water 53 (69.74%), butter and tea 5 (6.58%) and others (Table 2). This result implied that water contains the highest percentage of solvent or additives in the preparation of remedies. The local people reported that some of the additives used to improve the flavor and reduce adverse effects such as vomiting and diarrhea, so that the efficacy of the traditional medicine would be increased. A previous research study performed by [32] also reported such additives.

### 3.5. Conditions of Preparation from Plant Materials

The result of the study indicated that, the local people prepared the remedies from fresh, dry, and both fresh and dry materials. In this case, out of 193 preparations, 137 (70.98%) are in fresh form, 51 (26.43%) are dried, and 5 (2.59%) are both dried and fresh. The above data showed that the local people prepared the remedies dominantly from fresh materials. This might be due to the fresh medicinal plant part contents that are presented for a long period before use and effective to treat diseases in the study area compared to the dried form. Similar results obtained by [7, 23, 25, 35], and [8] showed that using fresh material was preferable than dry material for remedy preparation. The dependency of local people on fresh materials of the plant is a potential threat for the loss of these medicinal plants.

### 3.6. Route of Administration

Regarding the route of administration, oral 96 (49.74%) administration was reported as the most common route of administration followed by dermal 58 (30.05%) administration (Figure 4). This might be due to the reason that oral and dermal routes are more effective because the prepared medicines will react quickly with the physiology of pathogens and increase its curative power. The other reason is related with the presence of the wide spread of the internal diseases in the study area. This finding is agreed with some previous reports such as [25, 32], and [31] which indicated that oral was the most common route of administration.

### 3.7. Application of Prepared Remedies

The largest parts of prepared remedies are applicable by drinking 62 (32.12%) followed by eating 27 (13.98) and painting constituted 19 (9.84%) each and others (Figure 5). This result agrees with the work of [15, 22] in which drinking accounted the largest percentage of application of prepared remedies. Internal ailments were commonly treated by making the patient drink medication preparations; tooth infection was treated by crushing and applying the remedial plant part on the tooth surface; skin infections caused due to ringworms were treated by painting herbal preparations on the infected skin, and are applied on swollen body parts to cure swelling. Some plants do have different applications for different disease types. This preparation is used for different diseases by diverse application techniques.

### 3.8. Dosage Administered and Unit of Measurement

The effectiveness of healing particular human diseases is depending on the dosage of prepared medicinal plant. According to informants' response, the dose of plant remedies differed among traditional healers even in treating the same health problems. The plant remedies in the study area were prescribed with units of traditional dosage measurement such as Mankia (teaspoon), one hand, Fingal (coffee cup), Birchiko (teacup), Tassa (water cup), and Atiq (a third of finger length) which were commonly used. However, some prepared medicinal plants used by guessing (estimation) without being quantified by appropriate measuring instruments. About 52 (59.1%) of informants reported that the amount of dosage given to children and weak individuals are less than that of adults. However, measurements used to determine the dosages are not standardized. The amount of medicine prescribed by healers differs from place to place or from healers to healers and there is no standard dose as that of modern medicine [36]. According to [5], in most cases, the measurements are rough, lack precision, and dosage given to the patient has no strict specification. According to [37], the lack of precision is one of the shortcomings for the credit of the traditional healthcare system.

The majority of informants 62 (70.45%) reported that the medicine that they prepare and apply to treat the different health problems have no clear side effects on patients. Nevertheless, some of informants 23 (26.1%) have in fact informed noticeable side effects like vomiting, nausea, severe headache, diarrhea, gastric, burning wounded skin, loss of weight, and temporary unconsciousness that frequently occur while using medicinal plants against hepatitis, gonorrhea, wound, and rabies. Informants report temporary irritation on patients of hemorrhoids and skin infection. Pregnant women are also not given excess amount of medicinal plants that were poisonous to humans with observable adverse effects such as vomiting and diarrhea. This finding agreed with the finding of other studies by [38, 39].

### 3.9. Medicinal Plants Used to Treat Human and Livestock Diseases in the Study Area

A total of 89 medicinal plants were collected in the study area. Out of which 60 plant species (67.42%) were reported to treat the human diseases exclusively, 19 species (21.35%) were reported to treat both livestock and human diseases, and 10 species (11.23%) were reported to treat only livestock diseases. This result showed that the local people give more attention and have more traditional knowledge to treat human diseases than livestock diseases in the study area. Similar results were documented in other study sites of Ethiopia [15, 27, 28, 34], and [22].

#### 3.9.1. Medicinal Plants Used to Treat Only for Human Diseases

Medicinal plants that were collected in the study area that used for human health problems were 60 species. Among these 60 medicinal plant species, 54 genera and 33 families were recorded and identified. The family Fabaceae is the dominance family and constituted 6 species followed by Solanaceae which constituted 5 species, and Asteraceae constituted only 4 species. This result agrees with the work of [7, 8], which showed the dominance of family Fabaceae for the treatment of human diseases. However, dominance of family Asteraceae for the treatment of human diseases was reported in the work of [4, 15].

#### 3.9.2. Medicinal Plants Used to Treat Only for Livestock Diseases

Medicinal plants that are collected and identified in the study area used to treat livestock disease only are 10 species. They are grouped in 10 genera and 10 families. The total ten families constituted one species each. This result showed that only a few number of medicinal plant species are available as remedies for the treatment of livestock diseases as compared to the number of plant species used to cure human diseases. Furthermore, the local people have less traditional knowledge and practice to treat livestock diseases than human diseases in the study area. Majority of these medicinal plants are collected from wild vegetation. This result agreed with the work of [15] in which majority of medicinal plants were collected from the wild vegetation.

#### 3.9.3. Medicinal Plants Used to Treat Both Human and Livestock Diseases

Medicinal plants that are collected and identified in the study area used for both human and livestock health problems are 19 species. They are grouped in 18 genera and 16 families. Asteraceae constituted 3 species; Sapindaceae constituted 2 species; the rest of the family constituted one species each. Majority of these medicinal plants are wild. This result agrees with the work of [15] in which majority of medicinal plants were collected from the wild vegetation.

#### 3.9.4. Major Human Diseases and Plant Species Used to Treat Them

In the study area, totally 50 human diseases which were reported to be treated by 79 plant species (60 plant species treated only human diseases, 19 plant species treated both human and livestock diseases) were recorded. Some diseases were reported to be treated by more than one medicinal plant species and one medicinal plant species was reported to treat more than one human disease. Information from informants showed that stomachache is treated by 14 species; febrile illness is treated by 9 species; wound, evil eye, and eye diseases can be treated by 8 plant species each; common cold and skin rash are treated by 7 and 6 species, respectively. The rest of the diseases are treated by one to five medicinal plants. Indigenous knowledge of medicinal plant that treats more than one disease could be widely known (more popular) than the medicinal plant that treats only one disease. This is because of the fact that different people had the probability of getting indigenous knowledge and they use a particular medicinal plant to treat at least one common human ailment. Human ailment treated by more than one plant species can easily treated by local people. In a previous ethnobotanical study, for example, [4] reported 47 human diseases treated by 48 plant species, [21] reported 53 human diseases treated by 62 plant species, [27] reported 55 human diseases treated by 82 plant species, and [22] reported 44 human diseases treated by 50 plant species. Similarly, [31] found that stomachache can be treated by 14 medicinal plant species.

#### 3.9.5. Major Livestock Diseases and Plant Species Used to Treat Them

According to this study, in the Sedie Muja district, 17 livestock diseases treated by a total of 29 plant species (10 plant species treated only livestock aliments, 19 plant species treated both human and livestock aliments) were recorded. Like human ailments, more than one medicinal plant can treat livestock ailments and one medicinal plant can treat more than one livestock diseases. Eye diseases and wound were the leading, which were treated by 6 medicinal plant species, diarrhea followed by 4 species and the rest diseases are treated by one to three medicinal plants.

Number of medicinal plants used to treat livestock diseases are very less than medicinal plants used for the treatment of human diseases. This could be due to the reason that local people gave more attention (priority) to their own diseases than diseases of livestock and only medicinal plants subscribed to livestock's up on identification of diseases by symptoms. In addition, the respondents have limited knowledge about the treatment of livestock diseases compared to human ailments since livestock's lead sedentary way of life and residents are not pastoralists. Similarly, the related idea also reflected in other part of Ethiopia by [4] reported 34 livestock problems treated by 27 medicinal plants, [21] 17 livestock problems treated by 14 medicinal plants, [27] reported 14 livestock problems treated by 16 medicinal plants, and [22] reported 13 livestock problems treated by 3 medicinal plants.

### 3.10. Transfer of Medicinal Plants Knowledge

Currently, the local people of the study area that have indigenous knowledge of medicinal plants are older age generations. This could make the ethnomedicinal knowledge to be eroded due to the death of elderly knowledgeable members of the community. As most informants reported; modern medication, modern education, religious beliefs, and modernization (rapid changes in people's life style) contributed to the loss of indigenous knowledge of medicinal plants in the study area. A major problem observed at the study area was that very old age traditional healers kept their knowledge a secret, because they assume in such a way that the knowledge of medicinal plant is one means of income generating, and the healing power of the plant remedy decreases if the secret is out. In addition, traditional healers were locally said to be “Debtera'” and “Tenquay”. They were also called as “sir mash” (root excavators), and “kitelbetash'” (leaf cutter). Therefore, traditional healers had forced to keep their knowledge and practices in secret.

This study found that the main sources of traditional medicinal plant knowledge transfer are parents (56.8%) followed by elder son (18.2%), from relatives (11.4%), from religious book (9.1%) and others (4.5%) mostly descended orally (Figure 6). This oral transfer of knowledge without documentation ceases the knowhow of future generation about different traditional medicinal plant usage in the study area. Most respondents transfer their knowledge to their family. This means that most of the traditional knowledge of medicinal plant is passed along the family line. First-born children in the family are the main holder of responsibility in keeping the information and they are successor of their parents as well. Few others share the traditional knowledge to trustworthy and lovely neighbors and other blood relation persons.

### 3.11. Importance of Medicinal Plants in the Study Area

#### 3.11.1. Informant Consensus

The result of this study showed that all informants do not uniformly know medicinal plants. Some medicinal plants are more popular than others. This may be due to easy access, effectiveness of medicinal plant, and wider occurrence of disease to be treated. Among medicinal plants in the district, *Ruta chalepensis* is predominant to be cited by most of the informants 62 (70%) followed by *Ocimum lamiifolium* 59 (67%). This plant is widely used for the treatment of evil eye, febrile illness, and headache. *Ocimum lamiifolium, Allium sativum,* and *Euphorbia abyssinica* were placed 2nd, 3^rd^, and 4th ranks, respectively, in accordance with the number of informants citing. With this, other highly used medicinal plants mentioned by 8 or more informants, scoring percentage greater or equal to 9% are listed as shown in (Table 3). Similarly, study conducted by [23] in Debre-Libanos district, Central Ethiopia showed that *Ruta chalepensis* took the lead popularity followed by *Ocimum lamiifolium*. Acording to [40], the result implies that those listed medicinal plants with high informant consensus are important and could be prioritized for their pharmacological values.

#### 3.11.2. Informant Consensus Factor

The highest ICF value was obtained from diseases categories Evil eye (0.90) followed by abdominal pain, gastritis, and constipation (0.87). Common cold and cough showed relatively low ICF value (0.37) (Table 4). Unlike this, the study of medicinal plants in Debre Libanos showed common cold is the highest with ICF value of 89% [23]. The highest calculated ICF values indicate the best agreement among informants on the use of human medicinal plant species for treating a certain disease. Similarly, the study conducted by [15] in the Goma District, Jima Zone of Oromia Region showed that Evil eye had highest ICF value from disease categories. According to [2], high ICF values are important to identify plants of particular interest in the search for bioactive compounds.

#### 3.11.3. Preference Ranking

Analysis by preference ranking was carried out on seven selected medicinal plants, which were employed by key informants for the treatment of stomachache, common ailment of the district. Eight key informants were asked to give rank or order for those selected medicinal plants based on their degree of treating stomachache. The result of this study showed that *Euphorbia abyssinica, Otostegia intergrifolia,* and *Zingiber officinale* were ranked first, second, and third, respectively, based on its degree of treating stomachache. *Brassica nigra* and *Lepidium sativum* medicinal plants were used for stomachache treatment purpose though they were least preferred (Table 5). *Euphorbia abyssinica* was widely available in the study area. So, residents have been using this plant for treating stomachache. The study by [29] in the Berber district, Bale Zone of Oromia Region indicates that the preference ranking of medicinal plants used to treat stomachache showed that *Stephania abyssinica* was the most preferred one followed by *Solanium incanum*.

#### 3.11.4. Paired Comparison

A paired comparison was made to determine the most preferred medicinal plants among the five species that were used to treat febrile illness in the study area. The responses of 6 key informants showed that *Ocimum lamiifolium* ranked first followed by *Zehneria scabra* while *Clematis simensis*is the least favored over the other plant species cited in treating febrile illness (Table 6). A study by [22] in the Debark district, North Gondar and the result of paired comparison indicate that *Zehneria scabra* is much favored in treating febrile illness followed by *Otostegia intergrifolia.*

#### 3.11.5. Direct Matrix Ranking

The result showed that *Olea europaea* sub sp.*, Carissa spinarum,* and *Brucea antidysenterica* were ranked first, second, and third, respectively. *Calpurnia aurea and Ficus vasta* were medicinal plants that were used less for those stated under use categories (Table 7). *Olea europaea* sub sp. plant was available in the forest and home garden in the study area. The plant easily burnt for firewood and charcoal, and it was strong for furniture making and fencing, hence, it was preferred and widely used in the study area. The more utilized plant species (*Olea europaea* sub sp.) for multiple uses renders scarcity of species unless replantation, whereas least used species have a chance to be conserved. The result agrees with the work of [27] in the Ofla district, Southern zone of Tigray which indicates that *Olea europaea* sub sp. is the most widely used multipurpose medicinal plant.

#### 3.11.6. Fidelity Level Index

Analysis of percentage of informants claiming the uses of a certain plant species for the same major purposes could not be taken as the only criteria in proving the efficacious of plant species. Furthermore, fidelity level index could be calculated to see the medicinal use values of species. The medicinal plants that are widely used by the local people to treat one or very few ailments will have higher FL values than those that are less popular. In this study, *Allium sativum* and *Croton macrostachyus* were reported by many informants to treat evil eye and stomachache, respectively, though they have low value of informant consensus (Table 8). Hence, informant consensus could not be taken as the measure of the potential efficacy of medicinal plants in the fidelity level index analysis. For example, *Ruta chalepensis,* being reported by 70% of informants, with FL value of 0.37 is found to be the third species, next to *Allium sativum* (0.7) and *Carissa spinarum* (0.53) to treat evil eye.

### 3.12. Threats and Conservation Status of Medicinal Plants

People need plants for their daily life activity. This result showed that only a few number of medicinal plant species are available as remedies for the treatment of livestock diseases as compared to the number of plant species used to cure human diseases. The cause of threats to medicinal plants can be generally grouped into natural and human-induced factors. However, in the study area as reported by the informants, most of the causes for the threats to medicinal plant are the anthropogenic factors such as agricultural expansion, fire wood collection, fence, construction, and medicine. Some natural factors that are well known factors in the study area are drought and wildfire. To rank these threats of medicinal plants based on the degree of damage, seven key informants were selected for the preference ranking exercise for seven most threatening factors. Ranking of threats on medicinal plants (values 1–5: 1 is the least destructive threat and 5 is the most destructive one) was also conducted and values were summed up and ranks were given to each threat. According to informants' response in the study area, agricultural expansion scoring 32 was the most threatened factor followed by fire wood collection scoring 28 and charcoal scoring 25 (Table 9). A similar result was obtained by [21] in the Seru district, Arsi zone showed that agricultural expansion is the most threatened factor for medicinal plants. Moreover, the local people are highly dependent on the fresh leaves and roots of medicinal plants; these greatly threaten the medicinal plants, since there is no habit of preservation or storage of plant parts for later use [23].

Conservation of natural resources in general and medicinal plants in particular maximizes the benefit of creatures. This conservation practice whatever in-situ (in their natural habitat) or/and ex-situ (out of their natural habitat) has been practiced. The source of most medicinal plants in the district is wild (59.55%), so low conservation of wild medicinal plants cause scarcity. Though conservation approaches were not sufficient, people of the district have been practiced in variety of wise use aspects such as nursery sites: such site propagates and distributes various plant species to increase wealth of plant resource. Protected areas: mainly in mountains and religious practice centers in forests are protected and reserved. The reason why Churches and Mosques preferably harbor plant diversity is because, their thought prohibited to cut plant resources from these sacred groves. This possibly preserves both medicinal plants as well as indigenous knowledge. In the Sedie Muja district, patchy remnants of old-aged Afromontane forests that contain many medicinal plants can be found mainly around Churches and Mosques. According to [41] a study in the Farta district showed that no one tries to cut a single tree from churches because of the culture of the people. Forestation: the habit of replantation in every rainy season contributed for the wealth of plants since the deforested trees had been replaced. Terracing: widely practiced to protect soil erosion and increase plant growth. According to [42], conservation of medicinal plants in home garden is strategic and ideal.

## 4. Conclusion and Recommendations

### 4.1. Conclusion

Based on the result, it can be concluded that the study area is rich in diversity of medicinal plant species and largely from wild vegetation 53 (59.55%). People of the study area highly depend on medicinal plant resource for themselves and their livestock health care. Totally 50 ailments of human and 17 ailments of livestock were reported to be treated by traditional medicinal plants of the area. These also show the depth of indigenous knowledge and practice on medicinal plants to treat ailments. This indigenous knowledge of medicinal plants is owned by older age people.

It can also be concluded as herbs constitute the main source of traditional remedies followed by shrubs and tree species. Leaves were also found to be the most frequently used plant parts followed by roots for preparation of human and livestock remedies. The wide use of some medicinal plants, their various parts, and use of fresh plant materials leads to be the potential threats for the loss of medicinal plants in the study area. Medicinal plants mainly threatened by anthropogenic factors such as firewood collection, overgrazing, charcoal production, changing wild vegetation to farm land, and overpopulation have all been recognized as contributing factors to the loss of plant taxa. The oral-based knowledge transfer, refusal of young next generation to gain the indigenous knowledge, the influence of modern education, and lack of awareness were the major threats to vacant indigenous knowledge.

### 4.2. Recommendations

Based on the conclusions and findings of the study, the following recommendations are given:

- Local people should participate in cultivating medicinal plants in home gardens mixing with crops in the farmlands and live fences in addition to wild.
- We need to raise awareness to improve local community's knowledge on the importance, conservation, and management of medicinal plants largely to consider in-situ conservation of wild medicinal plants to ensure their sustainable use.
- The government should give recognitions and encourage the local herbal medicine practitioners to enhance the use of traditional medicine through licensing or certification and other incentives or by organizing them at community or district level, which popularizes their indigenous knowledge and medicinal plants use value.
- Training should be given to local people to have positive attitude toward traditional healers and to give prior emphasis to medicinal plants and multipurpose use tree species.

## Figures and Tables

**Figure 1:** Study area map.

**Figure 2:** Images of some medicinal plants with scientific name and corresponding local name recorded from the district.

**Figure 3:** Growth habit of medicinal plants in the study area.

**Figure 4:** Route of administration of medicinal plants in the study area.

**Figure 5:** Ways of application of medicinal plants in the study area.

**Figure 6:** Transfer of medicinal plants knowledge.

**Table 1:** List of medicinal plants used to treat only human diseases^∗∗∗^, only livestock diseases^*∗*^, both human and livestock diseases^*∗∗*^ in the study area: scientific name, local name, habit, habitat, disease treated, parts used, and conditions of preparation, method of preparation, dosage form, and route of administration.

No	Scientific name	Local name	Ha	Hab	Disease treated	Pu	Conditions, method of preparation and dosage	RA
1	Rumex nervosusVahl. ^*∗∗*^	Embaucho	S	Wd	Hemorrhoid	R	Fresh root is heated with fire and massaged the wound	D
					Snake bite	L	Fresh leaf is chewed and the solution is swallowed during the time of bite.	O
					Bone fracture	L	Fresh leaves are tied by threads on the affected part	D

2	Justica schimperiana (Hochst. ex Nees) T. Anders^∗∗∗^	Simiza	S	Bo	Stomachache	R	The fresh root is crushed and mixed with little water and then drunk	O
					Hepatitis	L	Fresh leaf is boiled with milk (decoction) and drunk with 1–3 cups of tea.	O
					Antrax	L + St	The shoot tip is cut, squeezed, and drunk by it mixing with a little water	O

3	Withania somnifera (L.) Dunal^∗∗∗^	Giziewa	S	Wd	Diarrhea	L	The fresh leaf is crushed, squeezed, and mixed with water and drunk	O
					Evil eye	R	The “Atik” size of dry root is cut, crushed and burnt in fire and fumigated.	F

4	Dodonaea viscosa L.f. ^*∗∗*^	Kitkita	S	Wd	Bone fracture	L	the fresh leaves are tied by treads on the affected part	D
					Evil eye	R	Dry root is covered with a piece of cloth and tied on the neck	D

5	Aloe Sp. ^∗∗∗^	Setie eret	H	Wd	Tinea versicolor	L	The fresh leaf is cut to isolate the fresh juice and creamed on the head	D
					Eye infection	L	Fresh leaf is squeezed and the juice is dropped on the eye	Oc
					Dandruff	L	The fresh juice is painted on the head	D

6	Zingiber officinaleRosco^∗∗∗^.	Zingible	H	Wd	Stomachache	St	Fresh stem is chewed and swallowed	O
					Common cold	St	Dry stem is pounded, boiled in tea, and drunk as one cup of tea	O
					Tonsillitis	R	Fresh root/rhizome is crushed and applied.	O

7	Phytolacca dodecandra L`Herit. ^*∗∗*^	Endod	S	Bo	Abortion	L	Fresh leaf is crushed, squeezed, mixed with water and one cup is drunk	O
					Malaria	R	The dry root or fresh root is pounded, powdered, mixed with water, and one glass cup is given to the patient	O
					Eye disease	L	Fresh leaf is crushed and mixed with butter then applied on the eye.	Oc

8	Plantago palmata Hook.f. ^*∗∗*^	Yewush milas	H	Hg	Abortion	R	Fresh root is crushed, squeezed, and mixed with water: the juice is isolated and 1–2 cups are drunk	O
					Toothache	R	Holding the fresh root (un processed) in between teeth.	D
					Bloating	L	Fresh leaf is crushed, mixed with water and given orally	O

9	Clematis simensis L. ^∗∗∗^	Azo hareg	Cl	Wd	Febrile illness	L + St	Fresh leaves and stem are boiled and fumigated	F
					Wound	L	Dry leaves are pounded, powdered, mixed with butter and applied on the wound	D

10	Xantium strumarium L. ^∗∗∗^	Chemud (Chegogot)	H	Wd	Eye infection	L	Fresh leaves are crushed, squeezed, and dropped on the eye	Oc
					Febrile illness	L	Fresh leaves are crushed and painted on the whole body part	D
					Acne	L	Fresh leaf is squeezed and applied to the affected skin. Three leaves are used for 7 days.	D
					Dandruff	L	The rubbed and squeezed fresh leaf is creamed on the head.	D

11	Ocimium lamiifolium L ^∗∗∗^	Damakesi	S	Hg	Febrile illness	L + St	Fresh leaves and stem are boiled with coffee and one cup is drunk	O
					Headache	L	Fresh leaf is crushed, mixed with water, and drunk.	O
					Diarrhea	L	Fresh leaf is boiled with tea and one cup of tea is drunk	O

12	Ficus vasta Forssk. ^*∗*^	Warka	T	Wd	Wound	L	Fresh leaf is crushed, squeezed, and creamed on the affected part.	D

13	Ruta chalepensi L.^∗∗∗^	Tena adam	H	Hg	Evil eye	L + St	Fresh leaves and stem are boiled with tea and one cup is given to patients	O
					Diarrhea	L	Fresh leaf together with salt (concoction) is chewed.	O
					Common cold	L	Fresh leaves are inhaled through the nose	N

14	Allium sativum L ^∗∗∗^	Nech shinkurt	H	Hg	Evil eye	Bu	Fresh bulb is eaten with injera	O
					Common cold	Bu	Fresh bulb is boiled with tea and one cup is drunk	O
					Malaria	Bu	Fresh bulb is crushed, mixed with honey, and soaked for seven days, then one spoon of the mixture is eaten in the morning for five days	O

15	Achyranthes aspera Lam.^∗∗∗^	Telenzh	H	Wd	Wound	L	Fresh leaf is crushed and tied on the wound	D
					Stomachache	R	Fresh root is chewed and swallowed during feeling of pain	O

16	Croton macrostachy us Del.^*∗∗*^	Bisana	T	Wd	Febrile illness	L + St	Fresh shoot tips are cut at seven areas of the plant and pounded, mixed with little water, and half cup is drunk	O
					Stomachache	R	Dry root is pounded, powdered, mixed with water, and one glass is drunk.	O
					Rabies	Ba	Dry bark is powdered and mixed with water and prepared with teff injera (concoction) and simply eaten	O
						Ba	Dry bark is powdered and mixed with water and 1 bottle is given orally	O
					Face fungus (tenea facie)	L + St	The fresh shoot tip is cut, squeezed, and the juice is applied on the face	O

17	Rhamnus prinoidesL. Herit. ^∗∗∗^	Gesho	S	Hg	Tonsillitis	L	Fresh leaves are crushed, squeezed, and put on the forehead	D
					Leishimaniasis	L	Fresh leaves are crushed and massaged on the wound.	D

18	Citrus limon (L.) Burm.f. ^∗∗∗^	Lomi	S	Hg	Tinea versicolor	Fr	Dry fruit together with egg is burnt and its ash is mixed with butter and then painted on the wound	D
					Skin rash	Fr	The juice of 1 fresh fruit is split, squeezed, and creamed on the skin.	D

19	Calpurnia aurea Ait (Benth). ^*∗∗*^	Digta	S	Wd	Gonorrhea	R	Fresh root is crushed, mixed with water, and one cup is taken for 3 days.	O
					Snake bite	R	Fresh root is crushed, mixed with water, and is given orally	O
					Diarrhea	L	The fresh leaf is crushed, soaked in water for 2–3 hrs, decanted, and one glass is administrated orally	O

20	Brucea antidysenterica J.FMill ^∗∗∗^	Abalo	S	Wd	Skin rash	L	Dry leaf is pounded, powdered, mixed with butter, and creamed on the skin	D

21	Buddleja polystachya ^*∗∗*^	Anfar	S	Bo	Wound	L	Dry leaf is pounded, powdered, mixed with butter, and painted on the wound	D
					Eyediseases	L	Fresh leaf is crushed, mixed with little water, and dropped on the eye	Oc

22	Capparis tomentosa Lam ^∗∗∗^	Gimero	S	Wd	Evil eye	R	Fresh root is crushed and sniffed through the nose	N
23	Carissa spinarum L ^*∗∗*^	Agam	S	Wd	Evil eye	R	Fresh root is crushed and sniffed through the nose	N
					Wound	R	Dry root is pounded, powdered, and applied on the wound.	D
					Diarrhea	R	Dry root is pounded, powdered, salt is added, it is made as a solution, and drunk	O

24	Sida schimperiana Hochst.ex.A. Rich. ^∗∗∗^	Chifrig	S	Wd	Stomachache	R	Fresh root is crushed, mixed with water, and one glass cup is drunk	O
					Evil eye	R	Fresh root is chewed	O

25	Cucurbita Pepo L. ^∗∗∗^	Duba	Cl	Hg	Tape worm	Se	Dry seeds are roasted, powdered, mixed with little water, and drunk	O

26	Eragrostis tef (Zucc.) Trotter ^*∗∗*^	Tef	H	Hg	Anemia	Se	Dry seeds are powdered, cooked, and eaten as a form of bread	O
					Lack of appetite and to fatten cattle	Se	Dry seeds are boiled, cooled down and then allowed to eat	O

27	Grewia ferruginea H ^∗∗∗^	Lenkuata	S	Wd	Retained placenta	L	Fresh leaf is crushed, squeezed, and half cup of tea is drunk	O

28	Lepidium sativum L. ^*∗∗*^	Feto	H	Hg	Stomachache	Se	Dry seeds are powdered, mixed with water, and drunk	O
					Febrile illness	Se	Dry seeds are powdered, mixed with a bulb of Allium sativum (concoction) and salt, and eaten.	O
					Diarrhea	Se	Dry seeds are pounded, powdered, mixed with water, and the solution has to be taken orally	O

29	Otostegia integrifolia Benth. ^∗∗∗^	Tinjut	S	Wd	Stomachache	L	Fresh leaf is chewed and swallowed	O
					Common cold	L + St	Dry or fresh leaf and stem together are burnt in fire and sniffed the smoke through the nose	N
					Devil/gine	L + St	Dry leaf and stem together are burnt in fire and fumigated	F

30	Cucumis ficifolius ARich. ^∗∗∗^	Yemidr enbuay	Cl	Wd	Stomachache	R	Fresh root is chewed and swallowed	O
					Snake bite	R	Fresh root is chewed and the liquid content is ingested	O

31	Rumex abyssinicus Jacq. ^∗∗∗^	Mekmeko	H	Wd	Skin rash	R	Fresh roots are crushed, mixed with water, and painted on the wound.	D
					Leishimaniasis	R	Fresh roots are crushed and tied on the wound using a clean piece of cloth.	D

32	Rosa abyssinica Lindley ^∗∗∗^	Kega	S	Wd	Devil	R	Dry root is burnt in fire and fumigated.	F
					Tapeworm	Fr	Handful of fresh ripened fruits (un processed) is directly eaten.	O

33	Impatiens tinctoria A. Rich ^∗∗∗^.	Ensosila	H	Hg	Rheumatic/arthritis	R	Fresh root is crushed and tied around the affected part	D

34	Tragia brevipes pax. ^∗∗∗^	Awulalit	Cl	Wd	Abortion	R	Fresh root is crushed, mixed with little water, and is drunk with half of coffee cup	O
					Evil eye	R	Dry root is burnt in fire and the smoke is allowed to enter the mouth	O

35	Crinum ornatum (L.f.ex Aiton) Bury^∗∗∗^	Yejib shinkurt	H	Wd	Tinea versicolor	R	Fresh root is crushed and creamed the content on the infected area.	D
					Ear disease	R	Fresh root is crushed, squeezed, and then its liquid is dropped through ear.	E

36	Euphorbia Schimperiana Scheele ^∗∗∗^	Anterfa	H	Wd	Male genital mutilation	La	The stem is cut to isolate the fresh latex and painted on the skin of tip part of the pines	D

37	Guizotia abyssinica (L. f.) Cass. ^*∗∗*^	Nug	H	Hg	Anthrax	Se	Dry seed is pounded, mixed with water and honey, and one glass cup is drunk	O
						Se	Dry seed is pounded, mixed with water, and given orally	O
					Febrile illness	Se	Dry seeds are roasted, pounded, mixed with water, and drunk	O
					Wound	Se	Dry seeds are chewed and applied on the wound	D
38	Echinops kebericho L.^*∗∗*^	Kebercho	H	Wd	Epidemics	R	Dry root is burnt in fire and fumigated	F
					Epidemics	R	Dry root is burnt in fire and fumigated	F
					Evil sprit	R	Dry root is powdered, burnt in fire, and fumigated	F

39	Brassica nigra L^∗∗∗^	Senafich	H	Hg	Stomachache	Se	Dry seeds are pounded, powdered, mixed with water, and eaten with injera	O

40	Verbena officinalis ^*∗∗*^	Atuch	H	Wd	Stop bleeding after birth	L	Fresh leaf is massaged and rubbed on the ear skin	D
					Wound	L	Fresh leaf is crushed, squeezed, and painted on the wound	D
					Diarrhea	L	Fresh leaves are crushed, mixed with water, and given orally	O

41	Aloe Sp. ^∗∗∗^	Wondie eret	H	Wd	Ear infection	L	Fresh leaf is crushed, squeezed, and the juice is poured into the ear canal	E

42	Clerodendrum myricoides (Hochst) R.Br.ex^∗∗∗^	Misirich	S	Wd	Swelling	L	Fresh leaves are crushed and pasted on the swelling	D
					Anthrax	L	Fresh leaves are squeezed and drunk	O
					Evil sprit	R	Dry or fresh roots are grounded with seeds of Allium sativum and leaves of Ruta chalepensis (concoction) powder are soaked in water and ingested.	O

43	Coriandrum sativum L. ^∗∗∗^	Dinblal	H	Hg	Cough	Se	Dry seed is powdered, mixed with honey, and two spoons of the mixture is eaten every morning until recovery	O
					Common cold	Se	Dry seeds are boiled with tea and drunk before meal	O

44	Linum usitatissimum L. ^*∗∗*^	Telba	H	Hg	Gastritis	Se	Dry seeds are boiled with sugar and cooled down then one glass cup is drunk every morning for ten days	O
					Retained placenta	Se	Dry seed is powdered and homogenized and mixed with water and boiled (decoction) and then the solution is drunk after being cooled.	O

45	Trigonella foenum Graceum L ^∗∗∗^	Abish	H	Hg	Constipation	Se	Dry seeds are powdered, soaked with water for 12 hours, filtered the fluid, added sugar and concoction, and drunk	O
					Rheumatic/arthritis	Se	Dry seeds are grinded, powdered, and homogenized in water and drunk with a spoonful.	O

46	Datura stramonium L^∗∗∗^	Astenagir	H	Wd	Tinea versicolor	L	Fresh leaf is crushed, squeezed, and painted on the head	D
					Ear infection	L	Fresh leaf is crushed, squeezed, and the sap is dropped into the ear canal	E
					Toothache	Se	Dry seed is roasted, powdered, burned in fire, and fumigated the smoke trough the mouth	F
					Fire burn	L	Fresh leaf is crushed, squeezed, and painted on the affected area	D

47	Coffea arabica L.^∗∗∗^	Buna	S	Wd	Cough	L	Fresh leaf is boiled and one cup is drunk at night for few days until recovery	O
					Wound	Se	Dry seed is roasted, pounded, powdered, and the powder is added to the wound	D
					Diarrhea	Se	Dry seed is roasted, powdered, mixed with honey, and one or two spoons is taken in the morning time for three days	O

48	Ziziphus spina christi. ^∗∗∗^	Geba	S	Bo	Wound	L	The fresh leaf is crushed, squeezed, and painted on the wound	D
					Tinea corporis	L	Fresh leaf is massaged and rubbed on the affected area	D
49	Saccharum officinarum L. ^∗∗∗^	Shenkor ageda	H	Hg	Cough	St	Fresh stem is crushed, squeezed, boiled and cooled down, and one cup of tea is taken at night for five days	O
					Gastritis	St	Fresh stem is chewed and the juice is swallowed during the time of pain	O

50	Capsicum annuum L.^∗∗∗^	Karia	H	Hg	Malaria	Fr	Fresh raw fruit is eaten with injera	O

51	Stephania abyssinic A. RICH ^∗∗∗^	Yeayt hareg	Cl	Wd	Hepatitis	R	Dry root is pounded, powdered, mixed with water, and half a glass cup is drunk	O
					Febrile illness	L + St	Fresh leaf and stem together are boiled and fumigated at night and the whole body is washed the next morning	F

52	Euphorbia abyssinica J. F. Gmel. ^∗∗∗^	Kulkual	T	Bo	Stomachache	La	The tip part is cut to isolate the latex, a drop of fresh latex is collected, half a cup is mixed with little water and drunk	O
					Malaria	R	Fresh root is crushed, mixed with water, and one coffee cup is taken	O
					Leshimaniasis	La	The fresh latex is applied on the wound until recovery	D
					Hemorrhoid	La	Fresh latex is painted on the wound	A

53	Artemisia afra Jack.ex willd. ^∗∗∗^	Chikugn	H	Wd	Devil	L + St	Fresh leaves and stem are crushed and sniffed through the nose	N
					Common cold	L	Fresh leaves are sniffed	N

54	Eucalyptus globulus Labill. ^∗∗∗^	Nech bahirzaf	T	Hg	Febrile illness	L	Fresh leaves are boiled, fumigated at night, and the whole body part is washed the next morning	F
					Common cold	L	Fresh leaf is boiled and sniffed through the nose	N

55	Alchemilla sp L^*∗∗*^	Lut	H	Wd	Abortion	R	Fresh root is crushed, mixed with water, and one cup is drunk	O
					Dandruff	R	Dry root is pounded, powdered, mixed with butter, and painted on the head	D
					To fatten calf and loss of appetite	R	Fresh root is crushed and mixed with water and then given orally	O

56	Jasminum grandiflorum L.^∗∗∗^	Yeset kest	S	Wd	Stomachache	L	Fresh leaves are chewed and swallowed	O
					Tetanus	Fr + L	Dry leaf and fruit are pounded, powdered, mixed with fresh butter (concoction), and creamed on the affected part.	D

57	Brassica carinata^∗∗∗^	Yehabesha gomen	H	Hg	Stomachache	Se	Dry seeds are pounded, mixed with water, and one glass cup is taken	O
					Chifie	Se	Dry seed is pounded, powdered, mixed with water, and then washed the body with the mixture	D

58	Cicer arietinum L ^∗∗∗^	Shimbra	H	Hg	Spider poison	Se	Dry seeds are powdered, mixed with water, and one glass cup is drunk	O

59	Solanum marginatum L.f^*∗∗*^	Geber Enbuay	S	Wd	Prevent pregnancy	Se	Seeds are simply swallowed	O
					Cough	Fr	Fresh fruit is squeezed, mixed with milk, and given orally	O

60	Foniculum vulgar Mill ^∗∗∗^	Ensilal	H	Bo	Arthritis	St	The fresh stem is crushed and painted on the affected area	D
					Dry cough/cough	L	The fresh leaf is crushed, soaked in milk, and one glass is drunk continuously.	O

61	Silene macrosolen Steud. ex. A. Rich ^∗∗∗^	Wogert	S	Hg	Evil sprit	R	Dry root is burnt with fire and fumigated	F
					Febrile illness	R	Dry root is pounded, powdered, burnt in fire, and the smoke is fumigated	F

62	Zehneria scabra (Linn.f.) Sondl. ^∗∗∗^	Hareg eresa	Cl	Hg	Febrile illness	L + St	Fresh leaves and stem are boiled, fumigated at night time, and washed the whole body early morning the next day	F
					Eye disease	L	Fresh leaves are boiled in water (decoction) and fumigated.	F

63	Myrtus communis L. ^∗∗∗^	Ades	S	Hg	Devil	L	Dry leaves are burnt in fire and fumigated	F
					Scabies	L	Dry leaves are pounded, powdered, and mixed with butter, and then applied on the affected area	D

64	Guizotia schimperi ^∗∗∗^	Adey abeba	H	Wd	Melasma	Fl	Flowers are collected, dried, pounded, mixed with water, and massaged the affected area	D

65	Artemisia absinthium L ^∗∗∗^	Aruti	H	Hg	Devil	L	Dry leaves are burnt in fire and fumigated	F

66	Physalis peruviana^∗∗∗^	Anbut (Awut)	H	Wd	Wound	Fr	Fresh fruit is squeezed and the sap of the fruit is added to the wound	D
					Fire burn	L	Fresh leaf is squeezed and then creamed on the affected part	D

67	Vicia faba L. ^∗∗∗^	Bakela	H	Hg	Boil	Se	Dry seeds are chewed and applied on the wound	O
					Leshmaniasis	Se	Fresh seed is chewed and put on the wound after scratching.	D

68	Tephrosia inerrupta Hochst. and Steud ex^∗∗∗^	Giramta	H	Hg	Mumps	St	Dry stem is covered with a piece of cloth and tied on the neck	D

69	Clausena anisata (Wild) Hook.f.ex.Benth ^∗∗∗^	Limbich	S	Wd	Menigitis	St	Dry stem is covered with a piece of cloth and tied on the neck	D
					Fire injury	L	Fresh leaves are crushed and tied on the injured area.	D

70	Millettia ferruginea (Hoshst.)Bak. ^∗∗∗^	Birbira	T	Wd	Skin rash	Fr + Se	Dry fruits and seeds are pounded, powdered, mixed with butter, and painted on the affected skin	D

71	Catha edulis Vahl) Forssk. ex Endl. ^∗∗∗^	Chat	S	Hg	Stomachache	L	Fresh leaves are boiled and one glass cup is drunk	O
					Evil sprit	L	Fresh leaves are chewed and put on the head of patients	D

72	Kalanchoe petitiana A. Rich. ^∗∗∗^	Andawula	H	Wd	Skin rash	L	Fresh leaves are put on the fire and the affected area is rubbed	D
					Tonsillitis	R	Fresh root is crushed, squeezed in the water, and one cup is taken orally.	O

73	Capsicum annuum L. ^∗∗∗^	Berberie	H	Hg	Prevent abortion	L	Fresh leaves are crushed, squeezed, mixed with water and drunk with one coffee cup	O

74	Argemone mexican^*∗*^	Nechlebash	H	Bo	Accident	R	Fresh root is crushed, mixed with water, and given orally	O

75	Inula confertiflora A. Rich^*∗*^	Woyina gift	S	Wd	Eye infection	L	Dry leaves are pounded, powdered, and applied the powder into the eye using a small bamboo tube	Oc
					Wound	L	Fresh leaves are crushed, squeezed, and the juice is dropped on the wound	D

76	Nicotiana tabacum L ^*∗*^	Tinbaho	H	Wd	Expel leech	L	Fresh leaf is crushed, mixed with water, and given orally	O
					Cough	L	Dry leaf is pounded and smoked as a cigarette through the nose	N
					Blackleg	L	Fresh leaf is crushed and given to livestock.	O

77	Premna schimperi Engl.^*∗*^	Chechiho	S	Wd	Eye infection	L	Fresh leaf is crushed and painted on the eyelid	Oc

78	Dodonaea angustifolia L.f^*∗∗*^	Ketetina	H	Wd	Expel leech	L	Fresh leaf is crushed, mixed with water, and given orally	O
					Hepatitis	R	Dry roots are burned on fire and smoke is inhaled through the nose.	N
					Rheumatic/Arthritis	R	Fresh roots are cut, washed, and then 5 pieces of roots are chewed with salt.	O

79	Schinus molle L. ^*∗*^	Kundo berberie	T	Hg	Bloating	L	Fresh leaves are crushed, squeezed, mixed with water, and given orally	O
					Eye diseases	Fr	Fresh fruits are chewed and spat into the eye	Oc

80	Momordica foetida ^*∗*^	Kura hareg	Cl	Wd	Wound	L	Fresh leaves are crushed and painted on the wound	D
					Febrile illness	L	Fresh leaf is crushed, mixed with water, and given orally	O

81	Juniperus procera^*∗*^	Yehabesha tsid	T	Wd	Febrile illness	L	Fresh leaves are simply eaten	O
					Antrax	L	Fresh leaves are crushed, mixed with water, and given orally	O

82	Plantago lanceolata L. ^*∗*^	Gorteb	H	Wd	Eye infection	L	Dry leaves are pounded, powdered, and the powder is added into the eye	Oc
					Wound	L	Fresh leaf is crushed and rubbed on the wound area	D

83	Ficus carica L^*∗∗*^	Beles	S	Wd	Ringworm	La	Fresh leaf is crushed to isolate fresh latex and creamed on the infected skin.	D
					Wound	La	Fresh leaf is crushed to isolate fresh latex and painted on the wound	D
					Hemorrhoid	La	The stem is cut to isolate the latex and the latex is painted on the wound	D

84	Acanthus sennii Chiov^*∗*^	Kusheshilie	S	Wd	Rabies	R	Fresh root is crushed and given with water to all animals.	O

85	Vernonia amygdalina Delile. ^*∗∗*^	Girawa	S	Wd	Bloating	L	Fresh leaf is crushed, mixed with water, and drunk	O
					Malaria	L	Fresh leaves are crushed, mixed with water, filtered, and drunk.	O
					Urinary problems	L	Fresh leaf is crushed with the leaf of Eucalyptus globulus (concoction), made into a solution, and then drunk.	O

86	Jasminium grandiflorum L. ^∗∗∗^	Tembelel	Cl	Wd	Eye disease	L + St	The fresh leaves and seven pieces of immature stems of Olea europaea are grounded, powdered (concoction), mixed with water, and 2–3 drops of the mixture are applied on the infected part for 3 days.	Oc
					Tape worm	L	Dry leaves are powdered and one spoonful of it is mixed with water and drunk per day to get relief.	O

87	Kanahia laniflora^∗∗∗^	Tifrena	S	Wd	Bleeding after delivery	R	Fresh roots are collected (un processed) and tied on the neck.	D
					Evil sprit	R	Fresh or dry roots are crushed with seeds of Allium sativum and leaves of Ruta chalepensis (concoction), powdered, soaked in water, and inhaled.	N

88	Olea europaea subsp. L.^∗∗∗^	Woira	T	Wd	Eye disease	St	Fresh stem with leaves of Jasminum abyissinicum are crushed, mixed with water (concoction), and 2–3 drops are applied on the eye.	Oc
					Tonsillitis	L	Washing the fresh juvenile leaf of Olea europea well to chewing and ingesting the juice.	O
					Toothache	St	The fresh stem is heated and caught between the teeth.	O

89	Pterolobiumstellatum (Fors) Brenan ^∗∗∗^	Kentefa	S	Wd	Stomachache	Ba	The fresh bark is chewed and swallowed	O
					Swelling	L	The fresh leaves are crushed and put on the affected part	D

Key : habit (Ha): (Herb (H); shrub (S); tree (T); climber (Cl)). Habitat (Hab): Hg = home garden, Wd = wild; Bo = both parts used (Pu); (B = bark, La = latex, Bu = bulb, R = root, L = leaf, Fr = fruit, Fl = flower, Se = seed, St = stem; L + St = leaf and stem together, Fr + L= fruit and leaf together; Fr + Se = fruit and seed together); Route of administration (RA): (O-oral, D-dermal, N-nasal, Oc-ocular, E-ear, A-anal, F-fumigate).

**Table 2:** Solvents and Additives used in medicinal preparation.

Additives	Frequency	Percentage
Water	53	69.74
Butter	5	6.58
Tea	5	6.58
Injera or bread	4	5.26
Honey	4	5.26
Salt	3	3.94
Coffee	1	1.32
Egg	1	1.32
Total	76	100

**Table 3:** Lists of medicinal plant species cited by more than 8 of informants (≥9%).

Medicinal plant species	Local name	Informants citing (^#^)	%
*Ruta chalepensis*	Tenadam	62	70
*Ocimum lamiifolium*	Damakesi	59	67
*Allium sativum*	Nechshinkurt	58	66
*Euphorbia abyssinica*	Kulkual	55	63
*Carissa spinarum*	Agam	52	59
*Zehneria scabra*	Haregresa	29	33
*Zingiber officinale*	Zinjible	25	28
*Croton macrostachyus*	Bisana	22	25
*Datura stramonium*	Astenagir	19	21
*Coffea arabica*	Buna	19	21
*Phytolacca dodecandra*	Endod	18	20
*Nicotiana tabacum*	Tinbaho	16	18
*Aloe* sp.	Eret	16	18
*Justicia shimperaina*	Simiza	15	17
*Xantium strumarium*	Chemud	15	17
*Calpurnia aurea*	Digita	13	15
*Echinops kebericho*	Kebercho	12	14
*Otostegia intergrifolia*	Tinjut	12	14
*Dodonaea angustifolia*	Ketetina	10	11
*Olea europaea*subsp.	Woyira	10	11
*Verbena officinalis*	Atuch	9	10
*Vernonia amygadalina*	Girawa	9	10
*Clerodendrum myricoides*	Misrich	8	9
*Alchemilla* sp.	Lut	8	9
*Plantago palmate*	Yewushamilas	8	9

**Table 4:** ICF for the given diseases category.

No	Category of diseases	Ns	Nur	ICF
1	Evil eye	8	72	0.9
2	Evil spirit and devil	11	24	0.57
3	Common cold, cough	13	20	0.37
4	Stomachache, gastritis, and constipation	17	119	0.86
5	Eye diseases, ear diseases, mumps, and meningitis	19	54	0.66
6	Fire burn, wound, toothache, headache, tonsillitis, tetanus, and anemia	29	51	0.44
7	Ascariasis, tapeworm, and diarrhea	13	46	0.73
8	Scabies, skin rash, ringworm, tineavesrsi, dandruff, and leshimania	21	54	0.62
9	Febrile illness and malaria	16	42	0.63
10	Hemorrhoid, anthrax, gonhrrae, arthritis, hepatitis, and swelling	17	27	0.38
11	Urinary problem, stop bleeding after delivery, prevent pregnancy, retained placenta, and abortion	11	23	0.55
12	Spider poison, snake bite, and rabies	7	16	0.6
13	Leech, black leg, bloating, and epidemics	12	30	0.62

Key : Nur: is the number of use reports from informants for a particular plant-usage category, Ns: is the number of species used by informants, and ICF: informant consensus factor.

**Table 5:** Preference ranking of medicinal plants used to treat stomachache.

Medicinal plant	Respondent (R)								Total	Rank
	R	R	R	R	R	R	R	R		
*Otostegia intergrifolia*	7	5	4	7	5	6	7	6	47	2
*Zingiber officinale*	3	7	6	6	4	5	5	5	41	3
*Brassica nigra*	2	2	2	1	3	4	4	2	20	6
*Lepidium sativum*	1	3	5	4	1	1	1	3	19	7
*Croton macrostachyus*	4	1	3	2	2	3	3	4	22	5
*Justica shimperina*	6	4	1	3	6	2	2	1	26	4
*Euphorbia abyssinica*	5	6	7	5	7	7	6	7	50	1

**Table 6:** Paired comparison of medicinal plants used to treat febrile illness.

Medicinal plant	Respondents (R)						Total	Rank
	R	R	R	R	R	R		
*Ocimum lamiifolium*	3	3	2	4	2	4	18	1
*Croton macrostachyus*	2	3	1	3	2	2	13	3
*Clematis simensis*	3	3	2	0	2	1	11	5
*Guizotia abyssinica*	1	2	3	3	0	3	12	4
*Zehneria scabra*	3	4	2	4	2	2	17	2

**Table 7:** Direct matrix ranking of medicinal plants with different uses.

Use	Medicinal plants					
	*Dodonaea viscosa*	*Brucea antidysenterica*	*Calpurnia aurea*	*Carissa spinarum*	*Olea europaea*sub sp.	*Ficus vasta*
	R	R	R	R	R	R
Med.	3	2	4	4	3	3
Food	0	0	0	3	0	0
Fen.	4	3	2	4	4	3
Fur.	0	2	1	1	4	1
F.W	5	4	2	3	4	4
Cha.	2	4	0	3	4	2
Cons	3	5	1	4	4	3
Fod.	4	3	0	2	3	0
Total	21	23	10	24	26	16
Rank	4	3	6	2	1	5

Key : Med. = medicinal, F.*W* = firewood, Fod. = fodder, Char. = charcoal, Cons. = construction, Fen. = fencing, Fur. = furniture.

**Table 8:** Fidelity level index for some plant species.

Disease	Plant species	Percentage of informants	Np	*N*	FL (Np/N)	FL (%)
Evil eye	*Ruta chalepensis*	70	21	57	0.37	37
	*Allium sativum*	66	14	20	0.7	70
	*Carissa spinarum*	59	9	17	0.53	53
Stomachache	*Justicashimperina*	17	11	26	0.42	42
	*Croton macrostachyus*	25	13	20	0.65	65

**Table 9:** Ranking of threats on medicinal plants.

Threats	Respondents (R)							Total	Rank
	R4	R13	R35	R33	R50	R71	R83		
Fire wood collection	3	4	4	5	5	4	3	28	2
Construction	4	4	2	2	3	3	3	21	4
Agricultural expansion	4	5	5	5	4	4	5	32	1
Fence	2	1	1	2	3	2	2	13	7
Drought	5	2	4	2	3	2	2	20	5
Fodder	2	1	3	1	4	3	2	16	6
Charcoal	4	3	3	4	3	4	4	25	3

## Data Availability

The data used to support the findings of this study are available from the corresponding author upon request.
